This article has been retracted.

# Evaluation Method of Comprehensive Quality of Environmental Protection Teachers Based on Big Data Analysis Technology

**DOI:** 10.1155/2022/6848352

**Published:** 2022-10-12

**Authors:** Wei He, Weijiang Zhou

**Affiliations:** Yuanpei College of Shaoxing University of Arts and Sciences, Shaoxing Zhejiang 312000, China

## Abstract

In order to improve the shortcomings that the weight of each index is easily affected by human influence in the evaluation of traditional teachers' comprehensive literacy, on the basis of the analysis of index coefficients, feature reorganization, and feature analysis, this paper constructs the comprehensive literacy of environmental protection professional teachers' education in the big data environment. The evaluation model is proposed, and a weight distribution scheme for teachers' comprehensive literacy evaluation indicators is proposed based on the hierarchical Bayesian beta-return model, so as to improve the rationality of the indicator distribution and make the prediction results more accurate. The simulation results further verify the superiority of the proposed model in improving the comprehensive quality evaluation level of environmental protection teachers.

## 1. Introduction

The century-old plan is education-oriented; the education plan is teacher-oriented. As the pioneers in the process of education reform, the teachers' professional quality improvement is the core of ensuring the quality of education [1]. We are in an era of globalization. With the continuous maturity of the Internet, big data, blockchain, and artificial intelligence technologies and their application in education, new types of procedural evaluations and diagnostic evaluations emerge as the times require [2–4]. Evaluation is the “bull's nose” and “baton” of educational development and will become the “steering wheel” of educational development. The development of education evaluation and talent evaluation has accumulated a lot of rich theories for us to learn from and use. Multiple intelligences theory, various talent theories, educational goal classification theory, cognitive diagnosis theory, nonintelligence factor theory, and brain science theory have been widely used in the field of educational evaluation and talent evaluation in western countries. These theories all show a common feature, that is, the evaluation of people is more and more a comprehensive and complex process. Evaluation issues are extremely complex and critical [5–7]. To cultivate a team of teachers with high comprehensive quality, we must fundamentally solve the problem of the baton of education evaluation. Therefore, evaluating teachers' comprehensive literacy through big data analysis can well solve some of the current problems. In this paper, an evaluation model of English teachers' educational ability under the big data environment is constructed, and a weight distribution model of English teachers' educational ability evaluation indicators is obtained based on the hierarchical Bayesian beta regression model.

## 2. Research Status of Big Data Analysis Methods

### 2.1. Basic Concepts of Big Data

From a macro perspective, big data links the physical world, information space, and human society [8–10]. The physical world is transformed into a big data reflection in the information space through technologies such as the Internet and the Internet of Things, and human society generates its own big data image in the information space by means of human-machine interfaces, mobile internet, and other means. For the information industry, big data has vigorously promoted the new generation of information technology industry (the new generation of information technology industry is built on the third-generation platform, mainly big data, cloud computing, etc.). From the perspective of socioeconomics, big data is the core connotation and key support of the second economy [11]. The concept of the second economy was proposed by the American economist author in 2011, that is, it consists of processors, linkers, sensors, actuators, and economic activities that run on them [12].

Compared with traditional data, big data has four basic characteristics (called 4 V characteristics in the industry), namely, huge data volume (volume), low value density (value), wide sources, diverse characteristics (variety), and growth rate (velocity). Among them, the diversity of data is the most important feature, which describes the nature of multisource heterogeneity of data. It can be seen that the core problem of big data is how to quickly obtain valuable information from a wide variety of data [13, 14].

Big data is usually inseparable from data mining, artificial intelligence, machine learning, etc. There are both connections and differences between these terms, which can be represented by a Piatetsky-Shapiro Venn diagram (Figure 1) [15]. Big data is often thought of as datasets that are beyond the capabilities of conventional software tools to capture, manage, and process as input for data mining, machine learning, and more. Machine learning is a core component of data science, employing techniques from computer science, statistics, and artificial intelligence to facilitate the automatic improvement of algorithms with experience. Data mining is defined as the specific application of algorithms to extract patterns from data, focusing on the application of the algorithm rather than the algorithm itself. Data mining is a process in which machine learning algorithms are used as tools to extract potential patterns of value in datasets. Deep learning is a process similar to data mining, which uses a deep neural network architecture and is a specific type of machine learning algorithm. The concept of artificial intelligence is relatively broad. It is a discipline about knowledge. It mainly studies how to represent knowledge and how to acquire and use knowledge [16]. Big data, machine learning, etc. are the foundations that support artificial intelligence.

### 2.2. Basic Process of Big Data Processing

The big data workflow analysis process is shown in Figure 2. Among them, data preparation and model building are the key tasks, the difficulty lies in data preparation, and the focus is on normative modeling. Data is modeled in terms of databases, data streams, data collections, and data warehouses. The magnitude of data and the diversity of data require data integration, cleaning, and filtering before processing to ensure follow-up work. The data preparation phase often encounters the problem of saturation of the analytical system. Therefore, the efficiency of data storage, filtering, migration, and retrieval must be considered when analyzing large-scale data.

### 2.3. The Main Research Direction of Big Data

According to the different focus of analysis, the related research on big data can be divided into two directions: (1) data processing and representation, mainly emphasizing the methods of collection, access, processing, and visualization; (2) statistical laws of data, focusing on microdata extraction of essential features and discovery of patterns. The collection, storage, and calculation of big data are mostly presented in the form of software tools, such as the Internet of Things and the Internet for data acquisition, the Hadoop Distributed File System and NoSQL database for data storage, and the Hadoop ecosystem for data computing, MapReduce, etc. Big data statistical analysis methods are largely the improvement and combination of various data analysis methods, including hypothesis testing, significance testing, etc. Data mining is also an important step and is used to probe large databases to discover unknown patterns or information. Deep mining of big data can achieve data classification, estimation, prediction, and other goals. After years of practice and exploration, the industry has become more and more aware that only coordinated and balanced development in two directions can ensure the steady growth and sustainable development of big data applications [17]. At present, the development focus of big data analysis is gradually transitioning from the technology of data processing to the science of data analysis.

### 2.4. Application of Big Data

As shown in Figure 3, big data was first used in business and financial fields and then gradually expanded to medical, energy, transportation, and other fields [18–21]. Among them, smart grid is one of the important technical fields of big data application. With the advancement of power informatization and the support of hardware systems such as smart substations, smart meters, and monitoring systems, it is possible to analyze smart grid big data. The data sources of the power grid mainly include electricity information acquisition system, wide area monitoring system, power distribution management system, and electric vehicle charging management system [22]. Among them, important research directions include socioeconomic status analysis, forecasting, demand side management/demand response, and power system transient stability analysis and control. IBM and C3-Energy developed a big data analysis system for smart grid, and Oracle proposed a public data model for smart grid big data.

Overall, the research on the evaluation method of teachers' comprehensive literacy is still in its infancy. Multisource heterogeneous characteristics, multisource data fusion technology, and heterogeneous data processing technology will become the direction of future research.

## 3. The Connotation of Teachers' Comprehensive Quality

### 3.1. Teacher's Morality and Virtue

The so-called teacher's morality and style refers to the professional ethics of teachers and their ideological and work styles, including teachers' professional ethics, professional spirit, ideas, and other aspects. Noble teacher morality and good teacher style are the inherent requirements of the special profession of teachers. Teachers are the mirrors of students' moral cultivation. A good teacher should take the law from the top, see the wise and think together, constantly improve moral cultivation, improve the quality of personality, and impart correct moral values to students.

### 3.2. Professionalism

Solid knowledge, excellent teaching ability, diligent teaching attitude, and scientific teaching methods are the basic qualities of teachers. Because education and teaching is a challenging, intelligent, and creative work, teachers need to have profound professional knowledge and scientific and cultural knowledge, and they need to constantly update their teaching concepts and knowledge structure and constantly improve their teaching level. We require students to master the basic knowledge and skills of the subject, to comprehend the thinking method of the subject, and to have the courage to explore and the innovative spirit and the practical ability to solve practical problems. Our teachers must first have higher requirements.

In the information age, a series of cross-cutting frontier issues have arisen, which puts forward new requirements for teachers, and it is necessary to cultivate compound teacher talents. Compounding is not just mastery of professional skills, but also the ability to apply intersecting knowledge to solve problems. This requires the teachers of the university to have a broad knowledge reserve and cannot be limited to the field of study. As a university teacher, in addition to professional knowledge in this field, they also need to understand multidisciplinary knowledge such as Chinese, English, politics, history, chemistry, physical resources, mathematics, society, psychology, art, and philosophy. A university teacher who teaches human anatomy should first know how to appreciate fine arts and painting, so that he can draw an accurate map of human tissues and organs; a teacher who teaches biochemistry and molecular biology should first understand organic chemistry and inorganic chemistry. Be able to explain the metabolic pathways of sugar, protein, and fat in the chemical reaction of the human body; a teacher teaching pathology should first understand the knowledge of histology and embryology, so as to guide students to compare the changes in the morphological structure of normal tissues and organs and diseased tissues and organs. Just imagine, if a medical university teacher does not understand physics, he can neither find the mechanism of external force in the case of spinal injury nor understand the basic principle of radiation therapy for tumors. University teachers must have a broad knowledge reserve, in order to be able to draw inferences from other facts in teaching, to elicit extensive references, to arouse classroom interest and enthusiasm for learning, and to teach students to learn thoroughly and masterfully.

### 3.3. Strong Scientific Research Ability

College teachers should coordinate scientific research and teaching well, use scientific research to drive teaching, and use teaching to promote scientific research. With the continuous innovation of medical technology in the information age, college teachers will also encounter some problems that cannot be explained by textbooks in the teaching process. Teachers should reflect, question, and ask questions to the extent that they are familiar with the existing knowledge, and trace the source one by one through scientific research practice, explore solutions, innovate practice, and understand the past and present and the ins and outs of knowledge. The latest achievements in scientific research can also be reflected in teaching activities. Through free and flexible application expansion, reform and innovation, and updating and reorganizing teaching materials knowledge, students' academic horizons can be broadened. Only when teachers coordinate scientific research and teaching well, will they have high-level scientific research results and high-quality teaching effects, and explore frontier and difficult issues in the field of discipline development. To engage in scientific research is not only to write project applications, formulate research plans, implement project research, and conduct seminars and exchange meetings, but the most important thing is to continuously learn, discuss, accumulate, and innovate in these processes, so as to cultivate the courage to explore rigorous and realistic scientific research. Attitudes are transmitted to students through teaching activities to improve the quality of personnel training.

### 3.4. Information-Based Teaching Methods

In today's internet era, the popularization of computers, tablets, and smart phones has made various information technologies one of the indispensable skills of college students, and the learning methods and learning scenarios of college students have undergone tremendous changes. Therefore, teachers cannot simply adopt traditional teaching methods to design teaching links but build a new teaching mode and learning mode according to the changes of the times. During the new crown epidemic, large-scale online teaching was carried out across the country, and teachers across the country used various information technologies to deeply integrate education and teaching, effectively promoting the development of intelligent teaching in the field of teaching supported by emerging technologies such as artificial intelligence, cloud computing, and virtual reality [23].

The development of intelligent teaching is supported by emerging technologies such as reality in the field of teaching. With the development of information technology, the traditional teacher-led classroom is gradually transformed into a student-centered intelligent classroom, and the interactive experience of teacher-student interaction, student-student interaction, and human-computer interaction will become the key link of teaching. Facing the reform of the education system, teachers need to continuously learn and master various information-based teaching software and platforms, such as MOOC, Xuetong, Classroom School, and Rain Classroom, relying on cutting-edge technologies such as information technology and artificial intelligence to integrate teaching resources and design teaching interaction, implementing intelligent teaching, and evaluating teaching effects [24].

### 3.5. Excellent Teaching Art

Teaching is an art, shaping the mind and delivering the spirit. The object of teaching is a variety of people with independent, complex, changeable thoughts, and characteristics. Teaching activity is not a one-way interpersonal activity but a two-way transfer and exchange of ideas, emotions, culture, and knowledge between teachers and students. The expression of language and the matching of manners are the keys to reflect the teacher's superb teaching art. Appropriate teaching methods are the way to realize the superb teaching art. Accurate, clear, fluent, humorous, and funny language can make the knowledge level logical and clear and guide students to grasp and understand knowledge simply and clearly.

Elegant and confident posture can make the classroom atmosphere infectious. And these also can attract students' enthusiasm and interest of learning. What's more, the use of various teaching methods such as question-based, heuristic, case-based which are based on information technology can present the knowledge interesting and concise, so that can guide students to become interested in the course and then extends to the enthusiasm of the course [2, 25]. This is the teaching art that university teachers need to have.

### 3.6. Advanced Spirit of Innovation

Innovation is the soul of the development of a country, a nation, an enterprise, and a school, and its essence is to emancipate the mind and make breakthroughs. Without innovation, there will be no development, no innovation, and no progress. Looking back at the five thousand years of history, from the four ancient inventions, to the modern industrial revolution, and then to the modern information age, the penetration of innovative thinking is inseparable. The development of the times and the progress of science and technology have brought about essential changes in people's ideas, and put forward new requirements for the level of university education in terms of depth and breadth, that is, focusing on the cultivation of talents' innovative thinking [3, 26]. As a university teacher who cultivates innovative talents, it should have innovative consciousness and innovative spirit. University teachers should maintain the desire and demand for information and knowledge acquisition, not stick to the traditional teaching mode, dare to question, be good at experimenting, have the courage to transcend in teaching and research, and constantly explore new ideas and methods for teaching and research. The future of the nation is crucial [27].

## 4. The Status Quo of Teacher Development in Colleges and Universities in My Country Based on Big Data

### 4.1. Insufficient and Perfect System and Mechanism for the Development of Higher Vocational Teachers

First of all, in most colleges and universities, because they have not established relatively sound systems and rules and regulations for cultivating outstanding talents, the organizational management system has been in a state of “absence.” An insufficiently sound management mechanism cannot train vocational teachers in an all-round way or promote their own development. Due to the lack of overall planning and top-level design for the development of teachers in vocational colleges, some vocational colleges are still in a relatively passive situation in cultivating outstanding teachers and staff. Secondly, colleges and universities have not invested a lot of funds in the direction of teachers' own development, so they have not established and established a sound guarantee mechanism, which has led to a serious lack of close communication between schools, departments, and teachers. The work of cultivating teachers in the school is incapable of continuing, and it does not help the school to create a good school spirit. Thirdly, the traditional and outdated evaluation mechanism is used, which is usually one-way evaluation or directional evaluation. This evaluation mechanism will directly lead to excessive demands on teaching results by college teachers, thus gradually ignoring the entire process of carrying out educational activities, making it difficult to improve and cultivate students' comprehensive literacy and comprehensive ability. Finally, my country's education is at a critical stage of development. In most colleges and universities, there is usually a serious lack of an effective reward mechanism. When teachers achieve excellent results, the lack of an effective mechanism for praise and incentives will also hinder teachers' initiative to improve their own abilities.

### 4.2. The Groups Covered by Teacher Development Are Not Comprehensive Enough

For most vocational colleges, it is a long process to improve teachers' own scientific research ability and practical teaching level. In this process, whether it is a senior and experienced teacher or a younger group of teachers, it is necessary to continuously update the basic professional knowledge system through continuous training and learning from beginning to end, so as to help teachers keep pace with the latest academic the frontier and progress together with the times. At this stage, most colleges and universities generally pay more attention to cultivating teams of young teachers. From different points of view, improving the comprehensive quality and comprehensive ability of young teachers is of great help and benefit to improving teachers as a whole, but this does not mean that improving young teachers' own teaching level can represent the group of teachers. Therefore, improving some groups does not mean to improve the overall ability. If the actual training needs of teachers at all levels are not really taken into account, the training of a certain group across the board will directly affect the sustainable and steady development of the professional group of teachers.

### 4.3. Lack of Professional Content Aimed at Cultivating Teacher Development

In most colleges and universities in my country, school-based training has always been one of the important measures to cultivate teachers' development. On the one hand, because the content of training is too broad, and the content focuses on experience guidance and practical teaching theory, there is a lack of practical training and no in-depth exploration of detailed issues, resulting in the development of teachers that cannot be targeted. On the other hand, the training topics carried out are relatively typified and similar [28]. Most colleges and universities have proposed “training for all staff,” but the universality of a large number of training topics that carry out full-staff training lacks stratification or classification. Guidance and training teacher development is not achieved overnight. The measures taken by college teachers at different stages are different, and the needs of training teachers for development are also different. From this, it can be seen that colleges need to put teachers at different stages. Sexual development needs are regarded as comprehensive development needs, which directly leads to the invisibility of the effectiveness of cultivating teacher development [29].

## 5. Model Building

Assessments are generally based on four broad categories of criteria: teaching, research, academic programs, and supporting organizational facilities and services, which form the main pillars of academic quality [30]. At the heart of the academic assessment process is the assessment of the teaching quality of individual courses/faculties by students taking the course. Under the traditional mode, the evaluation of teachers' educational ability mainly adopts the methods of setting teaching evaluation forms, reviewing textbooks, classroom teaching observation, and discussing evaluation results [31, 32]. In order to arrive at an evaluation result, some attributes (variables/indicators) inevitably need to be assigned weights. By changing the relative weights, it is possible to increase or decrease the importance of certain attributes that have a crucial impact on the outcome of the evaluation process for these attributes. In this case, the evaluation process itself becomes unreliable and easily subject to subjective factors.

In the large-scale network open course environment, the evaluation of teachers' teaching ability has the characteristics of openness and randomness [33]. Therefore, it is necessary to use quantitative mathematical model analysis methods to accurately evaluate the educational ability of university teachers, such as intelligent algorithms and big data processing technology. Evaluate and predict the educational ability of language teachers. Yu [34] conducted research on the improvement of teachers' teaching ability under the Internet “+” environment. Feng [35] put forward effective countermeasures to improve the teaching ability of college teachers from four dimensions: correct cognition of teaching ability, active participation in professional training, comprehensive innovation of teaching mode, and good after-class reflection.

### 5.1. Index Coefficient Analysis and Feature Recombination

Assume that the prior knowledge based on time series sampling in the statistical environmental protection teacher's educational ability evaluation coefficient data is expressed as {*x*_*i*_}_*i*=1_^*n*^. At the same time, it is assumed that the evaluation coefficient data has a linear correlation Gaussian process characteristic. Let the sequence of teacher educational ability evaluation coefficients be *y*_*n*_′, and the fitting model of the statistics-based teacher educational ability evaluation coefficient data can be expressed as follows:

(1) $$\begin{array}{c} x_{n}=\varphi_{0}+\overset{p}{\underset{i=1}{\sum }}\varphi_{i}x_{n-i}+\overset{q}{\underset{j=0}{\sum }}\theta_{j}\eta_{n-j}, \end{array}$$

where {*η*_*n*−*j*_} is a standard positive distribution with mean 0 and variance *σ*^2^; *φ*_0_, *φ*_1_, ⋯, *φ*_*p*_ is the time-reversed assessment of teachers' teaching ability; *θ*_1_, *θ*_2_, ⋯, *θ*_*q*_ are the average coefficients of the sliding time window; and *p* and *q* are the prior knowledge representation based on time series sampling and the number of sliding time windows, respectively.

In order to simplify the model, this paper assumes that the data distribution of teachers' teaching ability evaluation coefficients is calculated in a two-dimensional feature space. At the same time, the high-dimensional phase space reconstruction method is used to reconstruct the characteristics of teachers' teaching ability, and the multidimensional reconstruction is used to describe the performance attributes of teachers' teaching ability. The characteristic distribution matrix *L* of teachers' teaching ability can be described as follows:

(2) $$\begin{array}{c} L=\left[\begin{array}{c} \begin{array}{c} x_{1}^{T}\\ x_{2}^{T} \end{array}\\ \cdots \\ x_{N}^{T} \end{array}\right]=\left[\begin{array}{cccc} x_{1} & x_{1+\tau } & \cdots & x_{1+\left(m-1\right)\tau }\\ x_{2} & x_{2+\tau } & \cdots & x_{2+\left(m-1\right)\tau }\\ \vdots & \ddots & \ddots & \vdots \\ x_{N-1} & x_{N-1+\tau } & \cdots & x_{N-1+\left(m-1\right)\tau } \end{array}\right]. \end{array}$$

Among them, *m* is the correlation dimension of the feature information in the multidimensional teacher's teaching ability statistical data sequence; *τ* is the data sampling time delay; *N* is the number of data.

By combining formulas (1) and (2), the index coefficient analysis and feature reorganization of teachers' teaching ability evaluation can be realized, and further standard data input can be provided for the evaluation and prediction of teaching ability.

### 5.2. Characteristics

In the reconstructed *m*-dimensional feature matrix *L*, a sparse matrix of principal component distribution of teachers' teaching ability is constructed, and singular value points *L* = *U* · *S* · *C* are used to analyze teaching ability in big data environment. *U* and *C* are linear correlation matrices, expressed as follows:

(3) $$\begin{array}{c} C=\left\{c_{1},c_{2},\cdots ,c_{n}\right\}, \end{array}$$

where *n* is the number of elements in the linear correlation matrix *C*.

Further, the singular value of *L* is represented by *S*, and then the attribute set of big data eigenvalues is described as follows:

(4) $$\begin{array}{c} S=\mathrm{diag}\left(\sigma_{1},\sigma_{2},\cdots ,\sigma_{n}\right). \end{array}$$

Among them, *σ*_1_ > *σ*_2_ > ⋯>*σ*_*n*_ > 0.

Using any orthogonal matrix to remove the dimension of the original data of English teachers' teaching ability, the reconstruction moment *L* of the attribute feature set of teaching ability can be obtained. In the reconstructed matrix space, the big data analysis method can be used to perform cluster analysis on teachers' teaching ability data, and the reconstructed matrix of teachers' teaching ability indicators can be expressed as follows:

(5) $$\begin{array}{c} X=\left[\begin{array}{c} \begin{array}{c} x_{1}\\ x_{2} \end{array}\\ \cdots \\ x_{N} \end{array}\right]=\left[\begin{array}{cccc} a_{1}^{T}c_{1} & a_{N}^{T}c_{2} & \cdots & a_{1}^{T}c_{m}\\ a_{2}^{T}c_{1} & a_{N}^{T}c_{2} & \cdots & a_{2}^{T}c_{m}\\ \vdots & \ddots & \ddots & \vdots \\ a_{N}^{T}c_{1} & a_{N}^{T}c_{2} & \cdots & a_{2}^{T}c_{m} \end{array}\right]. \end{array}$$

Among them, x_i_(i ∈ (1, N)) is the *i*-th capability index, and *a*_*i*_^*T*^(i ∈ (1, N)) are the matrix coefficients.

## 6. Model Introduction

Based on the method of big data analysis, this section established a data fusion model for the evaluation index of teachers' educational ability and analyzes the fusion of hierarchical Bayesian and beta regression model [36] of the teaching evaluation index. A hierarchical Bayesian beta regression model was proposed. Next, the model was introduced in detail.

A random survey was conducted among school teachers and students when the sample data was collected, and *j* = 1, 2 represents two different sampling time periods. Let *n* = *n*_1_ + *n*_2_ be the total sample size, and *y*_*ij*_ denote the score given by the *i*-th assessor at time *j* (overall teaching/course assessment score). *X*_*ij*_ = (*x*_*ij*_, 1, *x*_*ij*_, 2, ⋯,*x*_*ij*_, *k*)^*T*^ represents the observations of *k* known attribute vectors. Without loss of generality, this paper assumed that all data have been normalized, that is, the values of all assessments are between (0, 1). To simplify the model, it was assumed that the data follows a beta distribution, that is, the mean of the data can be defined as the observed and unobserved attributes and a weighted linear combination of constant variance. Therefore, the coefficients of the model can be defined as weights, i.e., the addition of positive random variables.

For two different time periods (*j* = 1, 2), the model proposed in this paper was used for analysis, and its form was described as follows:

(6) $$\begin{array}{c} Y_{ij}\sim \text{Beta}\left(a_{ij},b_{ij}\right),\\ a_{ij}=\frac{\left(1-\mu_{ij}\right)\mu_{ij}^{2}-\mu_{ij}\sigma_{j}^{2}}{\sigma_{j}^{2}},\\ b_{ij}=\frac{\left(1-\mu_{ij}\right)\left(\mu_{ij}-\mu_{ij}^{2}-\sigma_{j}^{2}\right)}{\sigma_{j}^{2}},\\ \mu_{ij}=w_{j,1}x_{ij,1}+\cdots +w_{j,k}x_{ij,k}+w_{j,k+1}z_{ij}, \end{array}$$

where *μ*_*ij*_ represents the average of the response variable *Y*_*ij*_ (overall evaluation score) mean; *σ*_*j*_^2^ is the variance of the response variable; *W*_*j*_ = (*w*_*j*,1_, ⋯,*w*_*j*,*k*_, *w*_*j*,*k*+1_)^*T*^ is a random variable that measures the relative importance of different attributes and latent variables at time *j*. *z*_*ij*_ represents the assessment of rater *i*'s unspecified factor at time *j*, that is, an unobserved random variable.

Use the Dirichlet prior distribution, *W*_*j*_ ~ *D*(1,…,1) in weight processing. *σ*_*j*_^2^ obeys uniform prior distribution, namely *σ*_*j*_^2^~*U*(0, *m*), and *m* = mm{(1 − *μ*_*ij*_, *μ*_*ij*_)}. Furthermore, this article assumes that all variables are independent and come from a beta distribution with both parameters equal to 0.5.

## 7. Simulation and Analysis

During the simulation, a questionnaire survey was conducted on 95 students in the school to obtain the dataset. The structure, content, and selected topics of the questionnaire were determined by teachers with rich teaching experience (more than 20 years of teaching experience). Based on the principles of courseware teaching materials, examination process, teaching ability, high quality of teaching methods, and reasonable arrangement, some indicators are selected for the study. The indicators were shown as follows:

(1) Clarity of course objectives, (2) relevance of course content to course objectives, (3) relevance of course content to established standards, (4) the value of courseware, (5) the course content meets academic and professional requirements, (6) whether the course is completed or not, (7) the degree to which the examination subjects are compatible with the course content and teaching, (8) the degree to which the difficulty of the examination is compatible with the difficulty of the course, and (9) adaptability, (10) fairness and impartiality of exams, (11) curriculum preparation, (12) curriculum content excellence, (13) curriculum language organization, (14) teacher professionalism, (15) subject atmosphere and interaction, (16) fair treatment of students, (17) respect for students, and (18) overall teaching/course assessment score.

Figure 4 shows the comparison results of the indicator weights in two different time periods. In order to highlight the results of the weight changes of the indicators in different time periods, this paper used two indicators, the deviation and the posterior probability, for analysis, where the deviation refers to the difference between the two weight comparison results; the posterior probability *π*_0_ was to set the tail probability to zero, which is defined as the formula (7) shown

(7) $$\begin{array}{c} \pi_{0}=\min\left\{f\left(w_{1,l}-w_{2,l}>0\left|y\right.\right),f\left(w_{1,l}-w_{2,l}<0\left|y\right.\right),l=1,\cdots ,g\right\}, \end{array}$$

where *f*(.) is the tail probability density function.

As can be seen from Figure 4, when the zero value is in the center of the posterior distribution, the value of *π*_0_ is expected to be close to 0.5, indicating that there is no significant difference in the indicator weights between the two different time periods. When *π*_0_ is low (for example, below 5%), it can be concluded that there is a difference in indicator weights between two different time periods.

Further, Figure 5 presents the posterior statistical results of the indicators. It can be seen that the relative importance of the indicator of attribute number 15 is relatively high for students (the average posterior weight is about 14%), followed by the attribute number 9 (the average posterior weight is about 13%), and the attribute number 11 (the average posterior weight is about 13% and about 9%).

## 8. Conclusion

This paper used a hierarchical Bayesian beta regression model to evaluate and test the main components of teachers' teaching ability and quality. The coefficients of the model can be interpreted as weights, which are used to measure the relative importance of students to different attributes. Further, based on the big data analysis method, this paper established a data fusion model for the evaluation indicators of teachers' educational ability in environmental protection majors, so as to improve the rationality of index allocation and make the evaluation results more accurate. Future research directions include data cleaning and teacher ability evaluation under partial information problem to further improve the performance of the model.

## Figures and Tables

**Figure 1:** Venn diagram of important areas of data science.

**Figure 2:** Big data workflow analysis process.

**Figure 3:** Big data industry map.

**Figure 4:** Comparison results of indicator weights in different time periods.

**Figure 5:** Weighted posterior statistics.

## Data Availability

The dataset can be accessed upon request.
